# Comparison of Modular Control during Side Cutting before and after Fatigue

**DOI:** 10.1155/2021/8860207

**Published:** 2021-01-07

**Authors:** Naoto Matsunaga, Kenta Aoki, Koji Kaneoka

**Affiliations:** ^1^General Education Core Curriculum Division, Seigakuin University, 1-1 Tosaki, Ageo, Saitama, Japan; ^2^Waseda Institute for Sport Sciences, Waseda University, 2-579-15 Mikajima, Tokorozawa, Saitama, Japan; ^3^School of Sport Sciences, Waseda University, 2-579-15 Mikajima, Tokorozawa, Saitama, Japan; ^4^Faculty of Sport Sciences, Waseda University, 2-579-15 Mikajima, Tokorozawa, Saitama, Japan

## Abstract

The purpose of this study was to clarify the coordination between the trunk and lower limb muscles during sidestep and to compare this coordination before and after fatigue intervention. The intervention was lateral jump until exhaustion. Nonnegative matrix factorization (NMF) was used to extract muscle synergies from electromyography. Subsequently, to compare the muscle synergies, a scalar product that evaluates the coincidence of synergies was calculated. Three muscle synergies were extracted before and after the intervention from the NMF analysis. In accordance with the evaluation of the scalar product, these synergies were the same before and after the intervention. One of these synergies that engaged the internal oblique/transversus abdominis, rectus femoris, and adductor muscle was activated from before landing to midstance during sidestep motion; therefore, this synergy is thought to suppress excessive hip abduction. However, the activation timing of this synergy was delayed after the intervention (*P* = 0.028, effect size: 0.54, Wilcoxon test). This delay is considered to decrease hip stability. Thus, this change may induce a reduction in hip control function.

## 1. Introduction

Muscle synergy is defined as a group of muscle activities in synchrony and is extracted using mathematical methods, such as principal component analysis and nonnegative matrix factorization (NMF) [1]. In synergy analysis, electromyography is divided into two factors: (i) muscle synergy, which represents the relative weighting; and (ii) the time-varying component, which represents the relative activation of the muscle synergy [1]. Research on muscle synergy has been widely conducted in the fields of rehabilitation and neuroscience to evaluate activities of daily living, such as reaching tasks and locomotion [2–4]. In recent years, it has expanded to sports science and is expected to improve sports performance and prevent sports injuries [5–13].

Groin pain syndrome is common in soccer and rugby, wherein repetitive sidestep or side cutting motions are frequent [14–17]. It is defined as a dysfunction around the pelvis that results from poor mobility, stability, or coordination between the trunk and lower limbs, causing pain around the inguinal area [18]. Matsunaga et al. reported that the muscle synergies between the trunk and lower limb muscles during side cutting were different with and without groin pain [12]. However, whether the alteration of the synergy occurs because of groin pain or whether groin pain occurs because of the alteration of the synergy is unclear. In addition, groin pain is believed to be caused by overuse [14, 19, 20]. Overuse injury in sports occurs when the musculoskeletal structure receives a repetitive force, producing a combined fatigue effect over a period beyond the capacities of the specific structure [21, 22]. A previous study reported that the synergy changes due to transitory fatigue [11], and we hypothesized that it might be one of the risk factors for overuse injuries. Therefore, the purpose of this study was to compare the synergies during side cutting before and after transitory fatigue intervention. We hypothesized that the delay of the time-varying component will occur because the synergy time-varying component of the subjects with groin pain will be delayed.

## 2. Materials and Methods

### 2.1. Subjects

We recruited young healthy men with an exercise routine. Nine men (mean ± SD: age, 20.8 ± 2.2 years; height, 1.74 ± 0.06 m; and weight, 67.3 ± 5.7 kg) participated in this study. They had performed hard training as high school students and had been performing physical activities two to three times per week at the recreational level when they participated in this study. Their sports included soccer, badminton, baseball, and rugby. The exclusion criteria included a history of lower limb disorders that included groin pain syndrome, neurological disorders, or lower limb surgery. This study was approved by the ethics committee of our university (2010–270). All the subjects read and signed an informed consent form prior to participation.

### 2.2. Test Exercises

The test exercise was 5 repeated sidesteps with a width of 1.1 times the subject's height. The protocol was performed in the following order: first, five repeated sidestep motions at full effort, followed by the fatigue intervention, and finally, 5 repeated sidestep motions at full effort in the fatigue state. The subjects performed lateral jumps as a fatigue intervention. Lateral jumps can impose a large load on many muscles around the hip [23]. The width of the lateral jump was the same as the subject's height. The fatigue intervention required continuous lateral jumping, and fatigue was reached when the subjects could not keep jumping in sync with the metronome (DB-60, BOSS Co., Japan) rhythm at 60 Hz or jumping the distance of their height.

### 2.3. Data Measurement

To measure muscle activity, a wireless electromyography (EMG) system (EMG-025, Harada Electronic Co., Japan) was used. The activities of the following 8 muscles were measured as described by Matsunaga et al. [11]: rectus abdominal (RA), external oblique (EO), internal oblique/transversus abdominal (IO/TrA), erector spinae (ES), rectus femoris (RF), semitendinosus (ST), gluteus medius (Gmed), and adductor (ADD). All the muscles measured were on the right side. The RA electrodes were placed 3 cm lateral to the umbilicus. The EO electrodes were placed midway between the costal margin of the ribs and iliac crest, approximately 45° from the horizontal plane. The IO/TrA electrodes were placed approximately 2 cm medial and inferior to the anterior superior iliac spine (ASIS), and the ES electrodes were placed 3 cm lateral to the L4 spinal process. The RF electrodes were placed on the belly of the muscle corresponding to the center point between the ASIS and the upper margin of the patella. The ST electrodes were placed on the center point between the ischial tuberosity and medial epicondyle of the femur. The Gmed electrodes were placed 3 fingerbreadths from the lower region of the iliac crest. The ADD electrodes were placed 4 fingerbreadths from the lower region of the pubic symphysis. Before the surface electrodes were attached, the skin was rubbed with a skin abrasive and alcohol to reduce skin impedance to a level <2 k*Ω*. Pairs of disposable Ag/AgCl surface electrodes (Vitrode F-150S; Nihon Kohden Co., Japan) were attached parallel to the muscle fibers. The sampling frequency was set to 1000 Hz. To normalize the EMG data, a maximum voluntary contraction (MVC) test was performed on each muscle before the test exercise. The MVC for the RA was obtained, while the subjects performed a partial sit-up with their knees flexed and manual resistance was applied. For the EO, the subjects were in a supine position, with their knees and trunk flexed and rotated to the left. Resistance was applied to the shoulders, with the trunk extending and rotating to the right. For the IO/TrA, the trunk was instead flexed and rotated to the right, with the resistance applied at the shoulders, and the trunk extending and rotating to the left. For the ES, the MVC task was trunk extension performed in the prone position with manual resistance applied to the upper thoracic area without leg movement. For the RF, the subject sat on a chair with the hip and knee flexed to 90° and performed knee extension. Resistance was applied at the shank in the knee flexion direction. For the ST, the subjects performed knee flexion in the prone position, with the knee flexed to 45°. Resistance was applied at the shank in the knee extension direction. For the Gmed, the subject was in a side-lying position with the right side up and the hip extended and performed hip abduction with resistance applied in the hip adduction direction. For the ADD, the subject was in the side-lying position with the right side down with the hip extended and performed hip adduction with resistance applied in the hip abduction direction. Manual resistance was gradually increased up to the subject's limit and then held for 3 s.

Three three-dimensional motion capture cameras (Oqus, Qualisys, Sweden) were used to determine the timing of foot contact and push-off. The laboratory (global) orthogonal coordinate system (frame) followed the right-hand rule and had the positive *x*-direction orientated toward the left, the positive *y*-direction orientated toward the back, and the positive *z*-direction orientated vertically upward. To obtain kinematic data, reflective markers (QPM190, Qualisys, Sweden) were attached to 10 landmarks as follows: bilaterally on the edge of the toe on the shoes, the internal and external pastern on the shoes, the anterior superior iliac spinae, and 2 markers were placed on the floor, on either side of the subject. Kinematic data were collected at 200 Hz and synchronized with the EMG system.

### 2.4. Data Analysis

We analyzed the third round of sidestep motion during the test exercise. We determined the timing of landing using the acceleration of the edge of the toe marker. The EMG data were obtained from 200 ms before landing to 200 ms after push-off based on the kinematic data. A custom MATLAB (MATLAB R2016, MathWorks, Inc., Natick, MA, USA) code was used to analyze the EMG data. The raw data were band-pass filtered between 20 and 450 Hz and full-wave rectified. Then, they were interpolated to 200 time points. The EMG data were normalized relative to the associated MVC data of the muscle. As previously described, NMF was performed to extract modules [1], as follows:

(1) $$\begin{array}{c} \text{E}=\text{WC}+\text{e}\cdots \text{formula }1\\ \underset{\begin{array}{c} \text{W}>0\\ \text{C}>0 \end{array}}{\min}{\left|\left|\text{E}-\text{WC}\right|\right|}_{\text{FRO}}\cdots \text{formula }2, \end{array}$$

where *E* is a *p*-by-*n* initial matrix (*p* is the number of muscles and *n* is the number of time points). The initial matrix comprised normalized EMG data and a cycle for each of the 8 muscles; therefore, *E* is a matrix with 8 rows and 200 columns. *W* is a *p*-by-*s* matrix (*s* is the number of synergies) and represents muscle synergy, *C* is an *s*-by-*n* matrix and represents the time-varying component, and *e* is a *p*-by-*n* residual error matrix. Formula 2 indicates that matrix “*e*” calculated using formula 1 reaches a minimum. *W* is a vector; therefore, the calculated *W* is written as $\overset{⃑}{W}$. For each subject, we iterated the analysis by varying the number of synergies between 1 and 8, and then selected the least number of synergies that accounted for >90% of the variance accounted for (VAF) [5, 24, 25]. Global VAF was calculated based on the findings of previous studies.

(2) $$\begin{array}{c} \text{Global VAF}=\left(1-\frac{\sum_{i=1}^{p}\sum_{j=1}^{n}\;{\left(e_{i,j}\right)}^{2}}{\sum_{i=1}^{p}\sum_{j=1}^{n}\;{\left(E_{i,j}\right)}^{2}}\right)\times 100\;\left[\%\right]\cdots \text{formula }3, \end{array}$$

where *i* goes from 1 to *p* and *j* goes from 1 to *n*. Thus, *i* increases from 1 to 8, and *j* increases from 1 to 200 in this study. In addition, to confirm the reliability of our analysis, we also calculated the local VAF based on Hug et al. [24]:

(3) $$\begin{array}{c} \text{Local VAF }\left[m\right]=\left(1-\frac{\sum_{j=1}^{n}\;{\left(e_{m,j}\right)}^{2}}{\sum_{j=1}^{n}\;{\left(E_{m,j}\right)}^{2}}\right)\times 100\;\left[\%\right]\cdots \text{formula }4, \end{array}$$

where *m* represents the muscle. We defined the adoption standard for a local VAF >75% [24].

To compare *W* before and after the intervention, the scalar product (SP) was calculated based on the findings reported by Cheung et al. [4]:

(4) $$\begin{array}{c} \text{SP}=\frac{\vec{W_{\text{before}}}\times \vec{W_{\text{after}}}}{\vec{\left|W_{\text{before}}\right|}\left|\vec{W_{\text{after}}}\right|}\left(0≦SP≦1\right)\cdots \text{formula }5. \end{array}$$

The SP for the use of the correlation coefficients can assess the similarity of *W*. We defined the module as similar if the SP was above 0.75 [4].

In addition, to evaluate the level of fatigue, wavelet transform was performed based on the findings reported by Smale et al. [8], and the instantaneous mean frequencies (IMF) were calculated.

(5) $$\begin{array}{c} \text{IMF }\left(t\right)=\frac{\int \omega P\left(t,\omega \right)d\omega }{\int P\left(t,\omega \right)d\omega }\cdots \text{formula }6, \end{array}$$

where  *P*(*t*, *ω*) is the time-dependent power spectral density. After that, the IMF was averaged to calculate the mean frequency. The analyzed range of data was the same as that of the NMF analysis.

### 2.5. Statistics Analysis

Following the results of the Kolmogorov-Smirnov test, we used the Wilcoxon test to compare the mean frequency, peak timing of the time-varying component [7, 11], and muscle synergy weighting before and after fatigue using SPSS (ver 24.0, USA). The significance level was set at 0.05.

## 3. Results

Figure 1 shows the mean frequency of each muscle before and after fatigue. Among them, the mean frequency of the ADD decreased significantly (*P* = 0.036, effect size: 0.67).  Table 1 shows the relationship between the number of modules and global and local VAF. When 2 synergies occurred, the mean global VAF exceeded 90% for the first time. However, the mean local VAF did not exceed 75%. On the other hand, when 3 synergies occurred, the mean global and local VAF exceeded 90% and 75%, respectively. Therefore, 3 synergies were compared before and after fatigue in this study.

Figure 2 shows the extracted modules before and after fatigue. The SPs of modules 1, 2, and 3, which indicate the coincidence of muscle synergies, were 0.96, 0.97, and 0.86, respectively. For synergy 1, we found no significant difference in the peak activation timing (*P* = 0.909, effect size: 0.15). The activation timing of synergy 2 was significantly delayed after fatigue (*P* = 0.028, effect size: 0.54). Before fatigue, the activity of synergy 2 was observed in the first half of the sidestep sequence; however, it was seen in the second half after fatigue. The activation timing of synergy 3 did not differ before or after fatigue (*P* = 0.353, effect size: 0.36), and it occurred in the second half of the sidestep sequence. In addition, the weighting of ST decreased (*P* = 0.023, effect size: 0.54), while that of ADD increased significantly (*P* = 0.032, effect size: 0.54).

## 4. Discussion

This study investigated modular control during a sidestep sequence before and after fatigue. The results indicate that the synergies were similar before and after the intervention, and the main finding of this study was that the activation timing of synergy 2 was delayed after fatigue.

Muscle fatigue was confirmed using wavelet analysis. The spectrum shifts toward lower values if muscle fatigue occurs [26, 27]. In our study, the median frequency of ADD decreased significantly after fatigue. This result indicated that ADD was fatigued after the fatigue intervention.

The data from synergy 1 mainly reflected the Gmed and IO/TrA activities during the first half of the sidestep sequence. The activation level of synergy 1 gradually increased, and the peak activation was 25–35% of the sidestep sequence corresponding to the time of landing. The Gmed was the highest contributing muscle, and the IO/TrA and RF activities were also notable in this synergy. The extensor muscles of the lower limb began activating before landing to enhance joint stability and prevent injury. Therefore, it is theorized that synergy 1 functions in response to weight loads [11, 28–34].

Synergy 2 indicated coordination among IO/TrA, RF, and ADD. Before fatigue, this synergy was activated before landing until the middle stage of the sidestep sequence. It is considered that this synergy has a role in hip control because the hip abduction moment occurs after landing [11, 35]. In contrast, the activation timing of this module is delayed after fatigue. Matsunaga et al. [11] reported that synergy 2 is delayed in subjects with groin pain when compared with healthy subjects. Therefore, we believe that this timing delay may be related to the development of groin pain.

Synergy 3 engaged mainly the EO and ST and was activated in the last one-third of the sidestep sequence, corresponding to toe off. The EO contributes to trunk stability and ST activates hip extension. Therefore, synergy 3 is involved in the movement of kicking off the ground. In addition, the weighting of the ST decreased after fatigue, and the contribution of the ADD may show compensatory increases because the main function of the ADD is hip adduction, with hip extension being a supplemental function. The risk factors for groin pain are overuse [14, 19, 20, 36], dysfunction of the ADD [37–42], and hip stability [18, 43]. These reports indicate that compensatory ADD activity may influence the pathogenesis of groin pain.

This study had some limitations. First, our sample size was small. However, the results showed a sufficient effect size; therefore, we believe that the impact on the data in this study was small. In addition, we did not include women as our subjects because we attached devices on the unclothed upper body. This might have affected the sample size. Second, we could not perform a full motion analysis; therefore, we focused only on the timing of foot contact and toe off the ground to divide the sidestep into phases. Third, we did not judge fatigue using other methods.

## 5. Conclusion

We examined trunk and lower limb muscle coordination during the sidestep sequence and compared it before and after the intervention. As a result, the same 3 synergies were observed before and after the intervention. However, the activation timing of the synergy that functioned as a hip adduction control was delayed due to the intervention. This motor control deficiency may be related to groin pain syndrome and other injuries to the hip.

## Figures and Tables

**Figure 1:** Comparison of the mean frequency before and after fatigue. RA: rectus abdominis; EO: external oblique; IO/TrA: internal oblique/transversus abdominis; ES: erector spinae; RF: rectus femoris; ST: semitendinosus; Gmed: gluteus medius; ADD: adductor muscle. ^∗^Significant difference (*P* < 0.05).

**Figure 2:** Extracted synergies (left) and the activation pattern (right) during side cutting before and after fatigue. RA: rectus abdominis; EO: external oblique; IO/TrA: internal oblique/transversus abdominis; ES: erector spinae; RF: rectus femoris; ST: semitendinosus; Gmed: gluteus medius; ADD: adductor muscle. ^∗^Significant difference (*P* < 0.05).

**Table 1:** Relationship between the number of synergies and the global and local VAF. The number of synergies is decided when the global VAF exceeds 90% and the local VAF exceeds 75% for the first time.

		Number of synergies = 2		Number of synergies = 3	
		Pre	Post	Pre	Post
Global VAF (%)		91.8 ± 5.0	94.9 ± 5.3	96.4 ± 2.7	98.1 ± 1.8
Local VAF (%)	RA	35.2 ± 17.9	55.4 ± 40.0	81.1 ± 10.7	90.0 ± 12.2
	EO	64.6 ± 22.6	77.9 ± 16.9	86.5 ± 12.1	91.1 ± 10.1
	IO/TrA	54.6 ± 35.0	88.9 ± 10.1	95.6 ± 7.1	92.9 ± 7.9
	ES	69.0 ± 24.2	83.3 ± 19.7	88.3 ± 16.3	88.2 ± 11.9
	RF	50.7 ± 23.6	70.4 ± 17.4	89.8 ± 8.5	79.1 ± 15.4
	ST	48.9 ± 24.5	76.8 ± 25.7	86.7 ± 10.6	97.7 ± 3.9
	Gmed	44.4 ± 30.6	59.0 ± 34.1	88.7 ± 11.0	90.4 ± 12.2
	ADD	45.5 ± 24.5	69.7 ± 27.5	82.0 ± 13.4	88.7 ± 9.9

VAF: variance accounted for; RA: rectus abdominis; EO: external oblique; IO/TrA: internal oblique/transversus abdominis; ES: erector spinae; RF: rectus femoris; ST: semitendinosus; Gmed: gluteus medius; ADD: adductor.

## Data Availability

The data will be used in a future study.
